The article "Umbilical cord tissue-derived mesenchymal stem cells induce apoptosis in PC-3 prostate cancer cells through activation of JNK and downregulation of PI3K/AKT signaling" was retracted in 2018. Reason: lack of ethics approval or compliance.

# Umbilical cord tissue-derived mesenchymal stem cells induce apoptosis in PC-3 prostate cancer cells through activation of JNK and downregulation of PI3K/AKT signaling

**DOI:** 10.1186/scrt443

**Published:** 2014-04-16

**Authors:** Ihn Han, Miyong Yun, Eun-Ok Kim, Bonglee Kim, Min-Hyung Jung, Sung-Hoon Kim

**Affiliations:** 1 Cancer Preventive Material Development Research Center, College of Oriental Medicine, Kyung Hee University, 1 Hoegi-dong, Dongdaemun-gu, Seoul 130-701, Republic of Korea; 2 School of Medicine, Kyung Hee University, Seoul 130-701, Republic of Korea

## Abstract

**Introduction:**

Although mesenchymal stem cells (MSCs) have antitumor potential in hepatocellular carcinoma and breast cancer cells, the antitumor mechanism of human umbilical cord mesenchymal stem cells (hUCMSCs) in prostate cancer cells still remains unclear. Thus, in the present study, we elucidated the antitumor activity of hUCMSCs in PC-3 prostate cancer cells *in vitro* and *in vivo*.

**Methods:**

hUCMSCs were isolated from Wharton jelly of umbilical cord and characterized via induction of differentiations, osteogenesis, and adipogenesis. Antitumor effects of UCMSCs on tumor growth were evaluated in a co-culture condition with PC-3 prostate cancer cells. PC-3 cells were subcutaneously (sc) injected into the left flank of nude mice, and UCMSCs were sc injected into the right flank of the same mouse.

**Results:**

We found that hUCMSCs inhibited the proliferation of PC-3 cells in the co-culture condition. Furthermore, co-culture of hUCMSCs induced the cleavage of caspase 9/3 and PARP, activated c-jun NH2-terminal kinase (JNK), and Bax, and attenuated the phosphorylation of phosphatidylinositol 3-kinase (PI3K)/ AKT, extracellular signal-regulated kinase (ERK), and the expression of survival genes such as Bcl-2, Bcl-xL, Survivin, Mcl-1, and cIAP-1 in PC-3 cells in Western blotting assay. Conversely, we found that treatment of specific JNK inhibitor SP600125 suppressed the cleavages of caspase 9/3 and PARP induced by hUCMSCs in PC-3 cells by Western blotting and immunofluorescence assay. The homing of hUCMSCs to, and TUNEL-positive cells on, the K562 xenograft tumor region were detected in Nu/nu-BALB/c mouse.

**Conclusions:**

These results suggest that UCMSCs inhibit tumor growth and have the antitumor potential for PC-3 prostate cancer treatment.

## Introduction

Although clinical use of stem cells has been applied to various diseases, such as leukemia [1,2], Parkinson disease [3,4], diabetes [5], stroke [6], and cardiac disease [7-10], still limitations of their clinical use exist because of tumor-formation risk, host immune rejection, and ethical issues. However, mesenchymal stem cells (MSCs) are attractive compared with embryonic stem cells as a substitute resource for clinical use [11]. MSCs, also known as stromal progenitor cells, are found in several places in the human body, such as bone marrow, umbilical cord, umbilical cord blood, placenta, and muscle synovial membrane [12]. Under appropriate culture conditions, MSCs have the potential for self-renewal and differentiation into various cell lineages for osteocytes, adipocytes, and chondrocytes [13].

Recently, human umbilical cord blood (UCB) or human umbilical cord tissue mesenchymal cells (hUCMSCs), isolated from fetal origins, have been studied for clinical use because UCMSCs are considered to be a more-primitive precursor than MSCs [14,15]. Also, the umbilical cord matrix is suggested as a better source for the MSCs than umbilical cord blood in respect of higher expansion potential [16]. The hUCMSCs were known to express specific surface markers, such as CD44, CD105 (adhesion molecules), CD29, CD51 (integrin markers), SH2, and CD105 (mesenchymal stem cell markers), but not hematopoietic lineage markers, such as CD34, CD45, and HLA-class II [17-19]. Also, hUCMSCs have an immune-suppressive effect or reduced immunogenicity [20] and express vascular endothelial growth factor (VEGF) and interleukin (IL)-6 [18,21]. Recently, UCB-derived MSCs showed cytotoxicity against glioma [22] and Kaposi sarcoma [23], and umbilical cord mesenchymal stem cells suppressed the growth of breast cancer cells [24-26]. Based on previous evidence, in the present study, we investigated the antitumor mechanism of hUCMSCs in PC-3 prostate cancer cells and report that hUCMSCs induce antiproliferative and apoptotic effects in PC-3 cells via activation of JNK and inhibition of the PI3K/AKT pathway in either direct or indirect culture conditions.

## Materials and methods

### Culture for PC-3 prostate cancer cells and hUCMSCs

PC-3 prostate cancer cells were obtained from the American Type Culture Collection (ATCC, Rockville, MD, USA) and maintained in RPMI1640 containing 10% heat-inactivated fetal bovine serum (FBS) (Invitrogen, Carlsbad, CA, USA) and standard antibiotics (Invitrogen). In contrast, umbilical cord (UC) specimens were obtained within an hour of surgical resection under Kyung Hee Medical Center IRB-approved (KMC IRB 1125–03) just after appropriate written consent for the use of the human umbilical cord tissues.

Human UCMSCs were isolated from UCs of full-term delivery patients, as previously described [27]. In brief, UCs were washed in calcium, magnesium-free phosphate-buffered saline (DPBS), and cut into 1- to 2-mm^3^ pieces. Samples were enzymatically digested for 1 hour at 37°C with 3 mg/ml of collagenase type I (Sigma-Aldrich, St. Louis, MO, USA). Cells were filtered through a 40-μm nylon cell strainer and centrifuged at 1,500 rpm for 5 minutes, and pellets were collected as hUCMSCs. The cells were plated in 100-mm tissue-culture dishes at a density of 1 × 10^4^ cells/cm^2^ for growth at 37°C in a humidified 5% CO_2_ atmosphere in low-glucose Dulbecco modified Eagle medium (Invitrogen) with fibroblast growth factor (FGF)-2 (Sigma), insulin (Invitrogen), antibiotic solution (100 μg/ml penicillin, and 100 μg/ml streptomycin; Invitrogen), 1% gentamycin (Sigma), and heat-inactivated FBS (Invitrogen). Adherent cells were detached by incubation for 5 minutes with trypLE-Express (Invitrogen) and then replated at the same density.

### Osteogenic and adipogenic differentiation assays

Differentiation was induced according to established protocols [28]. In brief, for osteogenic differentiation, hUCMSCs were cultured to 80% to 90% confluency for 14 days in DMEM-LG supplemented with 10% FBS, 100 n*M* dexamethasone, 200 μ*M* ascorbic acid 2-phosphate, and 10 m*M* β-glycerophosphate. Alizarin Red staining was performed in subconfluent hUCMSCs for the visualization of calcium deposition. Cells were fixed with 4% paraformaldehyde for 10 minutes at room temperature, washed, stained with Alizarin Red staining solution for 1 hour in the dark, washed with 1 ml distilled water, and added by PBS. For induction of adipogenic differentiation, hUCMSCs were cultured to 80% to 90% confluence. Adipogenic differentiation media consisting of DMEM high glucose (Lonza) supplemented with 10% FCS, PSG, 10^−6^ *M* dexamethasone, 0.2 m*M* indomethacin, 0.1 mg/ml insulin, and 1 m*M* 3-isobutylmethylxanthine (Sigma-Aldrich) were changed twice a week for 14 days. The differentiated cells were fixed with 4% formaldehyde and stained with Oil Red O (Sigma-Aldrich) to visualize lipid vacuoles. The red lipid images were observed under phase-contrast microscope.

### Cytotoxicity assay

Cytotoxic effects of hUCMSCs against PC-3 cells were evaluated by 3-(4,5-dimethylthiazol-2-yl)-2,5-diphenyltetrazolium bromide (MTT) assay. We cocultured PC-3 cells by using Transwell assay system along with several densities of hUCMSCs for 24 hours in the same culture condition as hUCMSCs. The cells were incubated with 3-(4,5-dimethylthiazol-2-yl)-2,5-diphenyltetrazolium bromide (1 mg/ml) (Sigma Chemical Co., St. Louis, MO, USA) for 2 hours and then with MTT lysis solution overnight. Optical density (OD) was measured by using a microplate reader (Molecular Devices Co., Sunnyvale, CA, USA) at 570 nm. Cell viability was calculated as a percentage of viable cells cocultured with hUCMSCs versus single cultured control.

### Proliferation assay

DNA synthesis was detected by using a colorimetric bromodeoxyuridine (BrdU)-based Cell Proliferation ELISA kit (Roche Molecular Biochemicals, Mannheim, Germany) by following manufacturer’s instructions. In brief, we cultivated PC-3 cells by using Transwell assay system along with several densities of hUCMSCs in the same culture condition as hUCMSCs. For growing purposes, they were labeled with BrdU for 48 hours, as previously described [29]. The absorbance was measured at 450 nm by microplate reader (Tecan, Austria). Culture medium was used as a control for nonspecific binding.

### Immunoblotting analysis

Immunoblotting was done according to our standard protocols, as described previously [29]. The protein samples were extracted, quantified, and separated on SDS-PAGE gels and electro-transferred to nitrocellulose membranes. Nitrocellulose membranes were blocked in 5% nonfat milk and incubated with primary antibodies for PARP, BAX, Survivin (Santa Cruz Biotechnology Inc., Santa Cruz, CA, USA), cleaved caspase 9, Bcl-2, Bcl-xL, p-ERK, p-AKT, p-JNK (Cell Signaling Technology, Danvers, MA, USA) and β-Actin (Sigma). The blots were then exposed to HRP-conjugated secondary mouse or rabbit antibodies and analyzed by using enhanced chemiluminescence (ECL) Western blotting detection system (GE HealthCare Bio-Sciences, Piscataway, NJ, USA).

### Inoculation of PC-3 cells and hUCMSCs in mice

Nu/nu-BALB/c mice (4 to 5 weeks old) were purchased from the Shizuoka Laboratory Center (Kotoh, Japan) and maintained under classic conditions (55% relative humidity and 22°C ± 2°C). PC-3 cells and hUCMSCs were harvested and washed with 0.1 ml PBS. The cells gently were mixed with equal amount of growth factor-reduced Matrigel (BD BioSciences, San Jose, CA, USA) on ice. PC-3 cells (2 × 10^6^) were subcutaneously transplanted into the left flank of mice, and, 2 weeks later, hUCMSCs (5 × 10^6^) stained with PKH26 dye (Sigma) were transplanted into the right flank of mice. Eight weeks after PC-3 cell inoculation, Matrigel plugs were isolated from mice for H&E, immunohistochemistry, and TUNEL assay. The immunofluorescence staining image for PKH26 dye stained hUCMSCs in PC-3 cell tumor section was visualized under an Axio vision 4.0 fluorescence microscope (Carl Zeiss Inc., Weimar, Germany). This study was approved by and conducted in accordance with the policies set forth by the Animal Care and Use Committee of Kyung Hee University (Ref IRB; KHUASP(SE)-11–005).

### Terminal deoxynucleotidyltransferase dUTP nick-end labeling (TUNEL) assay

DNA fragmentation was analyzed by using Dead End fluorometric TUNEL assay kit (Promega, Madison, WI, USA). The tissues were fixed in 4% methanol-free formaldehyde solution in PBS for 35 minutes at 4°C and treated with terminal deoxyribonucleotidyltransferase (TdT) enzyme buffer containing fluorescein-12-dUTP for 1 hour at 37°C in the dark. The slides were mounted with mounting medium containing 4′,6-diamidino-2-phenylindole (DAPI) (Vector, Burlingame, CA, USA) and visualized under an Axio vision 4.0 fluorescence microscope (Carl Zeiss).

### Statistical analysis

Statistical analysis was performed by using Microsoft Excel analysis tools and SigmaPlot 2001 software. All data values are shown as means ± standard deviation (SD). The statistical significance was analyzed by using the Student *t* test and analysis of variance. *P* values of <0.05 were considered statistically significant.

## Results

### Characterizations of MSCs isolated from umbilical cord tissues

Regular morphology of isolated MSCs from umbilical cord (UC) was observed under phase-contrast microscopy, and very rare SA-β-gal-positive senescent cells were found in passages 0, 1, 3, and 5 of hUCMSCs by β-galactosidase assay (Figure 1A) [30]. As shown in Figure 1B, the normal proliferation rate of isolated MSCs was also confirmed (Figure 1B).

**Figure 1:** **Characterization of mesenchymal stem cells. (A)** Beta-galactosidase staining was used to check SA-β-gal activity in early passages (0, 1, 3, and 5) of hUCMSCs. Cell morphology was observed by phase-contrast microscopy. Scale bar, 50 μm. **(B)** Growth kinetics of the hUCMSCs according to the passages of hUCMSCs. **(C)** Characterization of isolated hUCMSCs was performed by identification of MSC markers, OCT4 (green) and NANOG (red). Nuclei were stained with DAPI (blue). Scale bar, 50 μm. **(D)** Characterization of isolated hUCMSCs cultured in adipogenic and osteogenic differentiation media for 14 days was performed by identification of the adipogenic and osteogenic differentiation assays, as described in Materials and Methods. The cells were stained with Oil Red-O and Alizarin Red dye staining, respectively. Scale bar, 100 μm.

Taken together, early passages of hUCMSCs are appropriate to use in this study. Porcine umbilical cord matrix cells express mesenchymal stromal markers and transcription markers such as OCT4, NANOG, and Sox [31]. Therefore, the expression of these MSC markers was evaluated in isolated hUCMSCs by immunostaining assay. As shown in Figure 1C, OCT4 and NANOG, which represent the pluripotent embryonic stem cell phenotype, were expressed in hUCMSCs. UCMSCs have multiple lineages potential to adipogenic and osteogenic differentiation [13].

To characterize the isolated hUCMSCs in our system, they were cultured in the adipogenic and osteogenic complete media. Ten days after induction, osteogenic differentiation of hUCMSCs was verified as brownish orange red for extracellular calcium deposits by Alizarin Red staining (Figure 1D, upper). In addition, accumulation of lipid vacuoles from the hUCMSCs as the indicator of adipogenic differentiation of MSCs was detected as bright red color by Oil-red staining (Figure 1D, lower), implying that isolated hUCMSCs in this study had stem cell potential.

### hUCMSCs inhibited the proliferation of PC-3 cancer cells

To determine the antitumor effect of hUCMSCs on human prostate cancer cells, PC-3 prostate cancer cells (1 × 10^5^) were cocultured with the densities of 3.33 × 10^4^, 2 × 10^4^, and 1 × 10^4^ of UCMSCs (hUCMSCs:PC-3 s ratio, 1:10, 1:5, 1:3). First, we determined the viability of PC-3 cells by MTT assay. The viability of PC-3 cells cocultured with UCMSCs (hUCMSCs:PC-3, 1:5, 1:3) was significantly decreased, whereas UCMSCs:PC-3 (1:10) did not show the difference compared with PC-3 cells cultured without hUCMSCs (Figure 2A). In addition, we determined the proliferation of PC-3 cells cocultured with hUCMSCs by BrdU assay. The growth of PC-3 cells cocultured with hUCMSCs was decreased to 44%, 49%, and 69% of control in the presence of UCMSCs with various numbers of 3.33 × 10^4^, 2 × 10^4^, and 1 × 10^4^, respectively, compared with untreated control (Figure 2B). As shown in Figure 2C, when PC-3 cells were cocultured in the presence of hUCMSCs (UCMSCs:PC-3, 1:3), the number of PC-3 cells was rarely observed compared with untreated control.

**Figure 2:** **The inhibitory effect of hUCMSCs on prostate cancer cell growth in direct or indirect coculture condition.** PC-3 cells (5 × 10^4^) were cocultured for 24 hours with or without hUCMSCs at ratio of 1:10, 1:5, and 1:3 (hUCMSCs:PC-3s). PC-3 cells were placed in the lower Transwell chamber, and different numbers of hUCMSCs (hUCMSCs:PC-3s, 1:10, 1:5, 1:3) were seeded in the upper chamber. **(A)** Effect of hUCMSCs on the viability of PC-3 cells by MTT assay. **(B)** Effect of hUCMSCs on the proliferation of PC-3 cells by BrdU assay. **(C)** Analysis of morphology of PC-3 cells cocultured with hUCMSCs by phase-contrast microscopy. **P < 0.01, ***P < 0.001 versus untreated control.

### hUCMSCs induced apoptosis and attenuated survival genes in PC-3 cells

To determine whether apoptosis is induced in PC-3 cells cocultured with hUCMSCs, Western blotting was performed. PARP cleavage, cleaved caspase 3, Bax, and phosphorylation of JNK were detected in the lysates of PC-3 cocultured with hUCMSCs (Figure 3A). To verify whether this apoptotic event is dependent on JNK pathway, the JNK-specific inhibitor SP600125 was treated in PC-3 cells cocultured with hUCMSCs. Conversely, the apoptotic features such as PARP cleavage, cleaved caspase 3, and phosphorylation of JNK in PC-3 cells by hUCMSCs were efficiently masked by JNK inhibitor SP600125 with Western blotting (Figure 3B) and immunofluorescence assay (Figure 3C). Also, as shown in Figure 4A, PI3K and phosphorylation of AKT and ERK were attenuated in PC-3 cells by hUCMSC cells. Furthermore, the expression of survival genes such as Bcl-2, Bcl-xL, Survivin, Mcl-1, and cIAP-1 was attenuated in PC-3 cells by Western blotting (Figure 4B).

**Figure 3:** **Effect of JNK SP60015 on PARP, cleaved caspase 3, cleaved caspase 9, and p-JNK induced by hUCMSCs in PC-3 cells. (A)** Effect of hUCMSCs on PARP, Bax, and cleaved caspase 9 in PC-3 cells. **(B)** Effect of JNK SP60015 on PARP, cleaved caspase 3, cleaved caspase 9, and p-JNK induced by hUCMSCs in PC-3 cells was detected in immunoblotting assay. **(C)** In the same condition as in **(B)**, expression levels of cleaved caspase, cleaved PARP, and p-JNK were analyzed by immunofluorescence assay. Each primary antibody was diluted 1/300. Light green indicates cleaved caspase 3, cleaved PARP, and p-JNK. DAPI (Blue).

**Figure 4:** **Effect of hUCMSCs on survival genes and JNK in PC-3 cells.** PC-3 cells were cultured for 24 hours alone or in the presence of hUCMSCs at the ratio (hUCMSCs:PC-3, 1:3). Cells lysates were immunoblotted with PI3K, p-AKT, AKT, p-ERK, ERK, p-JNK, JNK and PARP, Bax, cleaved caspase 9, and β-actin antibodies. **(A)** Effect of hUCMSCs on PI3K, AKT, ERK, and JNK in PC-3 cells. **(B)** Effect of hUCMSCs on Bcl-2, Bcl-xL, survivin, cIAP-1, and β-actin in PC-3 cells.

### The homing of hUCMSCs and apoptosis induction in PC-3 cells in nude mouse

Next, we investigated the homing of hUCMSCs to PC-3 cells in mice. PC-3 cells were injected subcutaneously into the left flank of the Balb-c/*nu-nude* mice. Two weeks later, PKH26-labeled hUCMSCs were transplanted into the right flank of the mice. Mice were killed 7 days after injection. Immunohistochemistry revealed that hUCMSCs were detected on the PC-3 tumor region with red color by confocal microscope (Figure 5A). In addition, TUNEL assay showed some TUNEL-positive cells in the PC-3 cancer cell region in mice treated with PKH26-labeled hUCMSCs (Figure 5B). However, we could not find a significant inhibitory effect of hUCMSCs on the growth of PC-3 cells for tumor weight and volume in mice compared with untreated control 3 weeks after PC-3 cell inoculation (data not shown). Thus, we must perform another animal study with a different number of hUCMSCs via direct or indirect injection of hUCMSCs into the PC-3 tumor region and check the possibility of teratoma in mice in the near future.

**Figure 5:** **Homing of hUCMSCs to PC-3 tumor site in Balb-c/*nu-nude *mice and their effect on TUNEL-positive cells in PC-3 tumor section. (A)** Paraffin sections for H&E and IHC staining with PKH26 dye (red). The PKH26-labeled cells tracking toward the PC-3 tumor region from the opposite-side flank. White arrows indicate the labeled PKH26 (red). **(B)** Representative photographs of TUNEL/PI staining. Red fluorescence (PKH26) marks transplanted hUCMSCs, and green indicates TUNEL-positive cells. DAPI (blue).

## Discussion

Mesenchymal stem cells (MSCs) are fibroblast-like multipotent stem cells that can be differentiated into several cell types, such as adipocytes, osteocytes, and chondrocytes [32,33]. MSCs are usually isolated from umbilical cord blood or tissues and adipocytes [34-36]. Although much evidence suggests that MSCs can be applied to several diseases, such as cancers [1,22,24], cardiac disease [8,37], stroke [6], and Parkinson and Huntington diseases [3], the underlying antitumor mechanism of MSCs was not fully understood until now. Thus, in the current study, the antitumor signaling of hUCMSCs was elucidated in PC-3 prostate cancer cells. We isolated hUCMSCs from umbilical cord tissues and confirmed positive stem cell markers, such as OCT4 and NANOG, and successfully induced osteogenesis by Alizarin Red staining and adipogenesis by Oil Red O staining, implying that hUCMSCs still have pluripotency of stem cells to be differentiated into adipocytes and osteocytes.

In addition, hUCMSCs treatment exhibited cytotoxic and antiproliferative effects in PC-3 cells by MTT and BrdU assays, indicating that hUCMSCs target the growth of PC-3 cells. Similarly, Khakoo *et al*. [23] supported that intravenously (i.v.) injected human MSCs home to sites of tumorigenesis and potently inhibit the growth of Kaposi sarcoma, and Chao *et al.*[24] reported that apoptosis was noted during coculture of MDA-MB-231 breast cancer cells with hUCMSCs. Furthermore, other groups reported that Z3-MSCs have an inhibitory effect on tumor growth by secretion of Wnt-inhibitor Dkk1, leading to downregulation of genes related to the cell cycle through inhibition of Wnt/β-catenin signaling [38,39]. Our results and other group reports mean that hUCMSC can be a potential therapeutic approach for the treatment of cancer. However, the ethical issues should be also considered, before we use hUCMSC as a therapeutic approach for tumor treatment.

In general, apoptosis, called programmed cell death, includes the intrinsic mitochondrial pathway and the extrinsic cell death pathway [40,41], and the activation of the JNK pathway is also related to apoptosis [42]. Here, hUCMSCs treatment resulted in the cleavages of caspase 9/3 and PARP, increased phosphorylation of JNK and upregulation of Bax as apoptotic protein, and decreased phosphorylation of PI3K/AKT and ERK in PC-3 cells by Western blotting, demonstrating the apoptotic effect of hUCMSCs via mitochondrial and JNK-dependent pathways. Consistently, hUCMSCs treatment attenuated the expression of survival genes, such as Bcl-2, Bcl-xL, Survivin, Mcl-1, and cIAP-1 in PC-3 cells, implying an inhibitory effect of hUCMSCs on antiapoptotic proteins.

To confirm the role of JNK in hUCMSCs-induced apoptosis in PC-3 cells, JNK inhibitor study was carried out. Conversely, treatment of JNK inhibitor SP600125 reversed the apoptotic ability of hUCMSCs to cleave caspase 9/3 and PARP in PC-3 cells by Western blotting and immunofluorescence assay, indicating that the JNK pathway mediates hUCMSCs-induced apoptosis in PC-3 cells. Consistent with our data, Aikin *et al.*[43] claimed that PI3K inhibition led to increased JNK phosphorylation and pancreas islet cell death, which could be reversed by the specific JNK inhibitor SP600125.

Of note, the homing of hUCMSCs to PC-3 cells and TUNEL-positive cells as an apoptotic feature was detected in the tumor section of PC-3 cells, implying that hUCMSCs on the left flank can move to PC-3 cells on the right flank, as the homing of hUCMSCs to PC-3 cells, possibly for cell death. Likewise, Liang *et al.*[44] reported that systemically infused hUCMSCs could home to the inflamed colon and effectively ameliorate colitis via modulation of IL-23/IL-17 by live *in vivo* imaging and immunofluorescent microscopy.

Overall, our findings demonstrate the antitumor potential of hUCMSCs for PC-3 prostate cancer treatment, but further study is required for animal tumor study via direct or indirect injection of hUCMSCs in the near future.

## Conclusions

Based on our results, UCMSCs inhibit the tumor growth and have an antitumor potential for PC-3 prostate cancer treatment.

## Abbreviations

ERK: Extracellular signal-regulated kinase; JNK: C-jun NH2-terminal kinase; PI3K: phosphatidylinositol 3-kinase; UCMSC: umbilical code mesenchymal stem cell.

## Competing interests

The authors declare that they have no competing interests.

## Authors’ contributions

IH: experimental design, data collection and participation in manuscript drafting. MY: design and conception for project, data analysis, manuscript drafting, and final approval of the manuscript. EK: acquisition and analysis of data and revision of manuscript. BK: partial data collection, revision of manuscript, and material support. MJ: revision of manuscript, experimental design, and material support. SK: design and concept, manuscript writing, and final approval of manuscript. All authors read and approved the final manuscript.
